# Optimization of Nanofiber Wearable Heart Rate Sensor Module for Human Motion Detection

**DOI:** 10.1155/2022/1747822

**Published:** 2022-06-16

**Authors:** Xiangbin Tang, Aihua Yang, Liangming Li

**Affiliations:** ^1^Institute of Physical Education, Hunan Normal University, Changsha 410012, China; ^2^Department of P.E, Changsha University of Science and Technology, Changsha 410017, China; ^3^School of Physical Education, Hunan University of Science and Technology, Xiangtan 411201, China

## Abstract

In order to further improve the detection performance of the wearable heart rate sensor for human physiological and biochemical signals and body kinematics performance, the wearable heart rate sensor module was optimized by using nanofibers. Nanoparticle-doped graphene films were prepared by adding nanoparticles to a graphene oxide solution. The prepared film was placed in toluene, and the nanoparticles were removed to complete the preparation of a graphene film with a porous microstructure. The graphene film and the conductive film together formed a wearable heart rate sensor module. The strain response test of the porous graphene film wearable heart rate sensor module verifies the validity of the research in this paper. The resistance change of the wearable heart rate sensor module based on the PGF-2 film is 8 to 16 times higher than that of the RGO film, and the sensitivity is better, proving that the sensor module designed by this method shows significant application potential in human motion detection.

## 1. Introduction

At present, there is a general upsurge in sports at home and abroad, with smart watches, sports bracelets, and smart phone sports software developing rapidly. But its function is relatively simple, it can only detect the body's exercise time, exercise distance, step length, stride frequency, number of steps, and heart rate during exercise. These indicators are not very helpful to the training of high-level athletes. With the development of nanotechnology and intelligent equipment, a real-time monitoring tool is made, which can monitor athletes' heart condition, breathing condition, and psychological reaction in different stages during training and can reflect athletes' exercise amount and intensity. During the exercise, the wearable heart rate sensor can evaluate the physiological signals and the performance indicators of the body kinematics during the exercise training process [1]. This sensor can be completely embedded and integrated in the athlete's smart bracelet, headband sweat band, sports clothing, and socks. Make this physiological monitoring enter a completely natural state. In recent years, scientists have explored many excellent physical and chemical properties of nanomaterials. The application of nanomaterials in the detection of disease markers has given birth to a series of ultrasensitive detection methods. The emergence of nanotechnology has opened new ways for ultrasensitive biosensors. Gold nanoparticles, graphene, carbon nanotubes, and DNA nanostructures have had an important impact on the design and development of biosensors [2–4]. As a result, some R&D institutions have developed some biosensors for doctors' diagnosis and patient disease monitoring. The development of these sensors has also attracted the attention of the sports world. It is believed that through these devices, coaches can obtain real-time sports data during athletes' training and record and analyze them. This resulted in the thinking about whether these smart devices can be used in the field of sports. This paper mainly studies the application of nanotechnology in the wearable heart rate sensor module. The sensitivity of the sensor is improved through the current nanofibers, so that it can more accurately monitor the physiological changes of athletes.

Nanotechnology and biotechnology are the two leading technologies of the 21st century, and there are many technological intersections between the two. In the past 20 years, the development of biosensing technology has been very rapid. It is a research field formed by the mutual penetration of many disciplines such as biology, chemistry, medicine, physics, and electronic technology. The new generation of nanotechnology biosensors developed by researchers from the Center for Applied Nanobiology and Medicine in the United States can see the reaction of human cells in specific microbes and different microbial components and see how these cells respond to certain drugs [5]. In later research, they will extend this technology to the field of sports to improve the sensitivity and specificity of the nanobiosensor for detecting some physiological and biochemical indicators of healthy humans. Zhu et al. [6] optimize the wearable heart rate sensor module, aiming at the existing wearable ECG and heart rate sensor BMD101, from the application level; it isolates the data channel, obtains a pure power source, and chooses the ECG electrode and the BMD101 sensor. The application and software design were discussed in depth, and various anti-interference optimization techniques were adopted to provide reference and reference for the design of wearable health monitoring microsystems. Zhang et al. [7] proposed a human motion tracking method based on wearable inertial sensors. This method comprehensively sorts out and summarizes the development history, research status, and typical methods of inertial human motion tracking technology, mainly including human kinematics models and biological constraints, sensor initial alignment methods, sensor types, sensor error processing, and data fusion methods, summarize the current status of the application of relevant methods in practice, and finally summarize the difficult problems to be solved in this field and carry out future development trends.

However, the sensors designed by the above two institutes are not ideal for human motion detection. Nanofiber wearable heart rate sensors can capture electrical signals from the human body, brain, and heart and output accurate and detailed human-related information after digital signal processing [8]. Coaches and athletes can use these products to monitor their physical and mental conditions during exercise, so as to more scientifically understand the physical condition of athletes during exercise and their adaptation to exercise intensity, monitor the exercise process, and improve the effect of exercise training. Therefore, this paper focuses on the detection of human motion and uses nanotechnology to optimize the design of the above-mentioned wearable heart rate sensor module. First, the preparation of graphene nanocomposite materials is studied. The thin film is placed in toluene to remove nanoparticles and prepare a porous microstructure graphene film; then, use graphene film and two layers of conductive film to complete the design of wearable heart rate sensor module, use the change of relative resistance to judge the response of the sensor module to strain, improve the sensitivity, and prove the practicality of the method in this paper through experiment sex.

## 2. Preparation of Graphene Nanocomposites

The choice of materials is also a very critical link in the realization of a wearable heart rate sensor, and graphene (GR) is a single-atom-thick carbon atom arranged in a honeycomb lattice, and it has been found to have special quantum dynamic properties, including “relativistic” electrons moving close to the speed of light, called massless Dirac fermions. Graphene has attracted widespread attention in recent years due to its excellent mechanical properties. Its fracture strain is about 25%, and Young's modulus is about 1.1 TPa, which makes it very suitable for the preparation of flexible and stretchable electronic devices [9]. In addition to excellent mechanical properties, graphene also has the following characteristics:

1. Good light transmittance, which can overcome the inherent performance limitations of traditional transparent electrode materials
2. Unique electrical properties, such as high carrier mobility and good piezoresistive sensitivity
3. Graphene is an ideal two-dimensional structural material, so it can realize the preparation of scalable devices through a top-down method and is compatible with existing manufacturing technologies [10, 11]

Graphene is a two-dimensional hexagonal lattice structure composed of a single layer of carbon atoms, but it is not a completely flat two-dimensional film, but there are a large number of microscopic undulations on its surface. Graphene is through this way to maintain its own stability. Graphene with a single atomic layer structure is the thinnest substance in the world, with an average thickness of only 0.34 nm; graphene has high hardness, and its Young's modulus reaches 1 TPa, and it has a breaking strength of 40 N^2^m^−1^, which is 200 of steel. At the same time, it has extremely high hardness, up to 300~400 N^2^m^−1^, elastic constant of 1~5 N^2^m^−1^, theoretical specific surface area value of 2600 m^2^g^−1^, and high charge mobility. These properties make graphene a good strain sensor material [12]. Therefore, a porous graphene film with better response to strain was prepared in this paper. By adding nanoparticles into the graphene oxide solution. Graphene films with physically mixed nanoparticles were prepared, and then, the nanoparticles are removed to obtain a graphene film with a porous microstructure [13, 14]. The responsiveness of the porous graphene film to strain was tested and applied to the test of physiological signals such as pulse and respiration. Design a wearable heart rate sensor module using the prepared porous graphene film [15].

### 2.1. Materials and Instruments

Table 1 shows the materials and instruments prepared by graphene nanocomposites:

### 2.2. Preparation of Porous Microstructure Graphene Film

#### 2.2.1. Handling of Slides

The slides were first rinsed with acetone three times, then rinsed with ethanol three times, rinsed with ultrapure water three to five times, and finally dried with nitrogen for use [16].

#### 2.2.2. Configure P(BA-Co-MMA)/Graphene Oxide Solution

Take 25 mg single-layer graphene oxide flakes in a 50 ml test tube filled with ultrapure water, and place it in an ultrasonic instrument for ultrasonic treatment for more than 6 hours to make the graphene oxide uniformly dispersed in the solution to obtain a 2 mg/ml graphene oxide solution. Take 4.17 mg and 6.25 mg of P(BA-Co-MMA) particles, respectively, into the solution; fully sonicate it to diffuse uniformly; and configure the mass ratio of P(BA-Co-MMA) particles to graphene oxide to be 1 : 4 and 1 : 6 solution [17].

#### 2.2.3. Preparation of Graphene Oxide Film Doped with Nanoparticles

Treat the glass slide obtained in the previous step with a vacuum plasma surface treatment machine for 5 minutes to make its surface hydrophilic. Use a pipette to suck 1 ml of the mixed solution prepared in the previous step, and apply it to the upper surface of the glass slide to make the solution spread evenly; and then, put it in a 60°C constant temperature drying oven for drying. Repeating the above dropping and drying steps can obtain graphene oxide films doped with nanoparticles of different thicknesses. A total of 10 times are carried out here to obtain a film with reliable mechanical strength [18].

#### 2.2.4. Reduction of Graphene Oxide Film

Place the nanoparticle-doped graphene oxide film adhered to the glass slide substrate in hydroiodic acid, heat it to 95°C, and keep it under this condition for 1 hour to fully reduce the graphene oxide to graphene [19–22]. After 1 hour, carefully pick up the film floating above the liquid surface, clean it thoroughly with ultrapure water, and soak in ultrapure water overnight (over 12 hours) to fully remove the hydroiodic acid residue on the graphene film.

#### 2.2.5. Remove P(BA-Co-MMA) Particles

Place the film prepared in the previous step in toluene, soak for 120 h to fully remove the P(BA-Co-MMA) particles in the film, and then, experiment with acetone, ethanol, and ultrapure water to fully clean it.

The preparation flow chart of porous graphene film is shown in Figure 1.

### 2.3. Strain Response of Porous Graphene Film

Use double-sided tape to paste the porous graphene film on the PI substrate, and then, fix its two ends on the vernier caliper, and change the degree of bending by changing the chord length of the arc formed by the bending. The reading of the vernier caliper is the chord length. From this, the radius of the circle formed can be calculated, and then, the strain of the graphene film can be calculated [15]. Suppose the chord length *c*, arc length *l*, center angle *θ*, and radius *r* are formed by the bending of PI base. Then, their relationship can be expressed as *θ*∗*r* = *l*; sin(*θ*/2) = *c*/2*r*, so the relationship between chord length and radius is *c* = 2*r*∗sin(1/2*r*). When the central angle formed by bending is *θl*, the corresponding radius is *r*_1_. Similarly, *θ*_2_ corresponds to *r*_2_. The bending strain can be expressed as *ε* = Δ*l*/*l* = [*θ*_2_(*r*_2_ + *z*) − *θ*_1_(*r*_1_ + *z*)]/[*θ*_1_(*r*_1_ + *z*)], and *z* is the distance from the center layer to the edge layer of the PI substrate. Because *r*_1_ > >*z*, *θ*_1_*r*_1_ ≈ *θ*_2_*r*_2_, so *ε* = *z*(*θ*_2_ − *θ*_1_)/*θ*_1_*r*_1_ = *z*(1/*r*_2_ − 1/*r*_1_). Because the original base is flat, *r*_1_ tends to be positive infinity, so *ε* = *z*/*r* = *h*/2*r* and *h* are the thickness of the base. The relative resistance change Δ*R*/*R*_0_ is used to judge the response of the wearable heart rate sensor module of porous graphene film to strain.

## 3. Construction of Wearable Heart Rate Sensor Module Based on Porous Graphene Film

The wearable heart rate sensor is composed of two layers of porous graphene film and two layers of conductive film. The conductive film is obtained by modifying the conductive polymer on the basis of the porous graphene film. The manufacturing process of wearable heart rate sensor is shown in Figure 2.

The specific assembly process is as follows: the prepared porous graphene film is cut into a 3 cm × 4 cm rectangle and then fixed on the base layer. The PPY-modified conductive layer is cut into a flag-shaped film with an effective area of 1 cm × 1 cm, and two cut conductive films are cross-stacked to form a sensor element with an area of 1 cm × 1 cm. Place the sensor element in the center of the base layer, and then, use silver paste to glue copper wires on the ends of the two flag-shaped films for later connection with the instrument for testing. Then, another porous graphene film is prepared on the sensing element. In this process, the other support layer and the encapsulation layer of the wearable heart rate sensor are prepared at the same time. After tailoring, a piezoresistive wearable heart rate sensor with a size of 3 cm × 4 cm is obtained. The wearable heart rate sensor uses a nanofiber substrate as a base layer, a sensing layer, and an encapsulation layer, respectively, and can be used for pressure response testing and human body motion detection.  Figure 3 shows the construction of a wearable heart rate sensor module:

## 4. Simulation Test

In this paper, PGF-1 porous graphene film prepared with 14.29% nanoparticles as pore template, PGF-2 porous graphene film, and RGO film prepared with 20.00% nanoparticles as pore template were, respectively, made into wearable heart rate sensor modules. Three membrane-supported modules were tested for strain response to verify the validity of this study. Respiratory rate and pulse are very important vital signs in medicine. The constructed sensor module is attached to a person's wrist or chest to record pulse and respiratory rate signals in real time. The experimental setup is shown in Figure 4.

The experimental device was attached to the wrist to detect the human body, and its stability and durability were tested first. Durability and stability are important parameters to measure the wearable heart rate sensor module. This experiment tests the stability of the wearable heart rate sensor module by repeatedly pressing the wearable heart rate sensor module under the condition that the external pressure is maintained at about 3 N, as shown in Figure 5. During the measurement process, the resistance signal and the pressing signal are exactly the same. In addition, the relative resistance values in the pressed state and the nonpressed state remained stable at 0.89 and 1, respectively.

Among them, (a) represents the response curve of the device after 600 compression cycles, and (b) represents an enlarged view of the partial data of the wearable heart rate sensor module of the porous graphene film in the compression cycle test. Analyzing Figure 5, it can be seen that the wearable heart rate sensor module of porous graphene film designed in this paper can withstand more than 600 compression cycle tests, and the performance of pressure sensing is not affected during the experiment.

Then, the strain response of the wearable heart rate sensor module made of three porous graphene films, namely, RGO film, porous graphene film PGF-1, and PGF-2, was tested, and the wearable heart rate sensor module of porous graphene film was obtained from a flat state. (40 mm) The test results when bent to a chord length of 37 mm are shown in Figure 6.

Figure 6 is the test result when the wearable heart rate sensor module with porous graphene film is bent from a flat state (40 mm) to a chord length of 37 mm. It can be seen from the figure that under the same stress conditions, three types of graphite the resistance of the wearable heart rate sensor module of the vinyl film have increased. This result indicates that the resistance of the three graphene films is very sensitive to the applied stress. When subjected to bending and stretching, the graphene sheets are stretched and misaligned, and the contact area becomes smaller, which causes the resistance of the wearable heart rate sensor module to increase. Compared with the RGO film, the resistance values of the porous graphene films PGF-1 and PGF-2 show significantly higher resistance changes under the same conditions, indicating that the wearable heart rate sensor module of the porous graphene film has a higher stress responsiveness which is more suitable for highly sensitive stress detection. This is mainly because the porous graphene film has a porous layered structure, and the graphene sheets have a wider variation space between the layers, so the relative resistance change is greater in the bent state. In addition, under the same stress conditions, the relative resistance change of the RGO film is about 8%, and the relative resistance change of the PGF-1 porous graphene film prepared using 14.29% nanoparticles as the pore template is about 17%. The relative resistance change of the PGF-2 porous graphene film prepared by using 20.00% nanoparticles as the pore template is about 46%. This result shows that the wearable heart rate sensor module using graphene film with more pore structure can achieve higher sensitivity for human motion detection stress. However, experimental results show that using more than 20.00% of nanoparticles as a pore template, it is impossible to prepare a complete porous graphene film. This is mainly because a small amount of graphene flakes cannot form a uniform film on the surface of the nanoparticles. Therefore, in this paper, we choose PGF-2 porous graphene film to design a wearable heart rate sensor.

The relative resistance changes of the wearable heart rate sensor modules made of three porous graphene films, RGO film, porous graphene film PGF-1, and PGF-2, under different bending states, are shown in Figure 7.

As shown in Figure 7, in the bending and stretching state, the resistance values of the three graphene film sensors all show an increase, and the resistance values of the wearable heart rate sensor modules of the three graphene films increase with the increase of stress and increase. This result indicates that the wearable heart rate sensor module of graphene film can quantitatively detect the applied stress. In addition, under the same bending and stretching conditions, the resistance value of the wearable heart rate sensor module of the PGF-2 porous graphene film is 8-16 times larger than that of the RGO film, indicating that the constructed porous graphene film is wearable. The heart rate sensor module has a more sensitive stress detection capability.

The gauge factor (GF) is usually used to represent the sensitivity of a strain sensor. It can be calculated according to (Δ*R*/*R*_0_)/Δ*ε*, and *ε* refers to strain. Convert the abscissa to the corresponding strain by *ε* = *h*/2*r*, and perform linear fitting. The result is shown in Figure 8.

The slope of the straight line indicates the strain response capability of the graphene film. Under different stretched states, the resistance change of wearable heart rate sensor modules based on PGF-2 film is 8 to 16 times higher than that of RGO film. When the strain is between 0.25% and 0.75%, the GF values of RGO, PGF-1, and PGF-2 strain sensors are 8.96, 122.08, and 282.28, respectively. This result shows that the constructed porous graphene film wearable heart rate sensor module has higher sensitivity and is more suitable for motion detection of weak physiological signals such as respiratory rate and pulse.

## 5. Conclusion

Wearable nanobiosensors can evaluate the physiological and biochemical signals and body kinematics performance indicators of athletes during training. This sensor is completely embedded and integrated in the athlete's clothing and can monitor the whole process of sports. During exercise, there is no need to connect any external equipment, making this physiological monitoring into a completely natural state. Develop the implantation of smart sensors in textiles. The fabric link integrates all the sensors on the clothing, so that each sensor type has its own typical reflection method. It can not only detect sweat composition and control exercise intensity but also feed back body movement in real time. It monitors the athlete's psychological state and provides a basis for scientific training. At the same time, its potential other functions will also be revealed. The structural materials used in the nanofiber wearable heart rate sensor module designed in this paper are all prepared from porous microstructured graphene films. Experiments show that the PGF-2 porous graphene film wearable heart rate sensor module designed in this paper has better stability than RGO, and the PGF-2 strain sensor prepared in this paper can withstand 600 times of pressing, and its resistance value is 8~16 times larger than RGO films. When the strain is between 0.25% and 0.75%, the PGF-2 strain sensor has the highest GF value of 282.28, which is superior to the contrast sensor and exhibits better sensitivity to small pressures, which makes it excellent in human motion detection. The transfer-type pressure sensor device was developed in the following research. Although the experimentally prepared biocompatible porous graphene nanofiber membrane has skin-friendly and breathable properties, it has poor water solubility and cannot be used to prepare transfer-type devices. In subsequent studies, we may consider fabricating devices by electrospinning using water-soluble polymers.

## Figures and Tables

**Figure 1:** Flow chart of preparation of porous graphene film.

**Figure 2:** The production flow chart of the wearable heart rate sensor.

**Figure 3:** Construction of a wearable heart rate sensor module.

**Figure 4:** Experimental setup.

**Figure 5:** Sensor cycle stability test.

**Figure 6:** Repeatability test results of strain response.

**Figure 7:** Relative resistance changes of porous graphene film pairs under different bending states.

**Figure 8:** Strain response.

**Table 1:** Materials and instruments prepared by graphene nanocomposites.

Material	Status	Material source
Single-layer graphene oxide	Flake	Nanjing Xianfeng Nano Material Technology Co., Ltd.
Absolute ethanol	Concentration 98%	Sinopharm Chemical Reagent Co., Ltd.
Acetone	Concentration ≥ 99.5%	Sinopharm Chemical Reagent Co., Ltd.
Methanol	Concentration ≥ 99.5%	Sinopharm Chemical Reagent Co., Ltd.
Ethyl acetate	Concentration ≥ 99.5%	Sinopharm Chemical Reagent Co., Ltd.
Dichloromethane	Concentration ≥ 99.0%	Sinopharm Chemical Reagent Co., Ltd.
Ammonia	Concentration 25% ~28%	Sinopharm Chemical Reagent Co., Ltd.
Acetaldehyde	Concentration 40%	Sinopharm Chemical Reagent Co., Ltd.
Deionized water	Resistivity ≥ 18	Lab homemade
Ultrasound system	SK250H	Kedao Ultrasonic Instrument Co., Ltd.
Electric heating constant temperature drying oven	DHG-9245A type	Shanghai Yiheng Technology Co., Ltd.
Scanning electron microscope	6500F	JEOL Company
Semiconductor characteristic analysis tester	Type 4200	Keithley Company

## Data Availability

The datasets used and/or analyzed during the current study are available from the corresponding author on reasonable request.
